The article "Why Hospital Pharmacists Have Failed to Manage Antimalarial Drugs Stock-Outs in Pakistan? A Qualitative Insight" was published in 2013. Journal: Malar Res Treat.

# Why Hospital Pharmacists Have Failed to Manage Antimalarial Drugs Stock-Outs in Pakistan? A Qualitative Insight

**DOI:** 10.1155/2013/342843

**Published:** 2013-10-07

**Authors:** Madeeha Malik, Mohamed Azmi Ahmad Hassali, Asrul Akmal Shafie, Azhar Hussain

**Affiliations:** ^1^Discipline of Social and Administrative Pharmacy, School of Pharmaceutical Sciences, Universiti Sains Malaysia, 11800 Minden, Penang, Malaysia; ^2^Hamdard Institute of Pharmaceutical Sciences, Hamdard University, F-8 Markaz, Johar Road, Blue Area, 4400 Islamabad, Pakistan

## Abstract

*Purpose*. This study aimed to explore the perceptions of hospital pharmacists towards drug management and reasons underlying stock-outs of antimalarial drugs in Pakistan. *Methods*. A qualitative study was designed to explore the perceptions of hospital pharmacists regarding drug management and irrational use of antimalarial drugs in two major cities of Pakistan, namely, Islamabad (national capital) and Rawalpindi (twin city). Semistructured interviews were conducted with 16 hospital pharmacists using indepth interview guides at a place and time convenient for the respondents. Interviews, which were audiotaped and transcribed verbatim, were evaluated by thematic content analysis and by other authors' analysis. *Results*. Most of the respondents were of the view that financial constraints, inappropriate drug management, and inadequate funding were the factors contributing toward the problem of antimalarial drug stock-outs in healthcare facilities of Pakistan. The pharmacists anticipated that prescribing by nonproprietary names, training of health professionals, accepted role of hospital pharmacist in drug management, implementation of essential drug list and standard treatment guidelines for malaria in the healthcare system can minimize the problem of drug stock outs in healthcare system of Pakistan. *Conclusion*. The current study showed that all the respondents in the two cities agreed that hospital pharmacist has failed to play an effective role in efficient management of anti-malarial drugs stock-outs.

## 1. Introduction 

Efficient drug management is the key strategy in reducing costs of drugs and ensuring their availability in the healthcare facilities [1]. High incidence of drug stock outs is diverse and imitates perpetual problems including inadequate resources and weak healthcare systems to delineate procurement needs and manage stock flows [2]. The selection of most cost-effective essential drugs to treat commonly encountered diseases, appropriate quantification, preselection of potential suppliers, procurement and monitoring of the performance of suppliers and the procurement system can be achieved by adopting efficient procedures. Failure in any of these areas leads to lack of access to appropriate drugs and waste of resources. Lack of properly trained staff in good procurement practices at key positions can also doom any procurement system to failure. Low incentives, inadequate posts, and lack of career development tend to confine potentials to attract and retain qualified staff in the healthcare facilities [3].

The article "Why Hospital Pharmacists Have Failed to Manage Antimalarial Drugs Stock-Outs in Pakistan? A Qualitative Insight" was published in 2013. Journal: Malar Res Treat.

Medicines procurement is an effective way to supply right medicines at right price to the patients in the healthcare facilities. No public or private healthcare system in the world can afford to purchase all drugs circulating in the market within its given limited resources due to these choices that have to be made [4]. The concept of nationally developed formulary or selection based on the essential drugs has been introduced in both developed and developing countries' healthcare systems to concentrate resources on the most cost-effective and affordable drugs to treat prevailing health problems. A limited list of drugs for procurement, based on an essential drugs list or drug formulary, defines which drug will be regularly purchased and thus is one of the most effective ways to control drug expenditures in the healthcare facilities [5].

The availability of antimalarial drugs recommended in the national essential drug list can be a measure of assessing how well malaria control is being implemented in reality. Acute shortage of artemether/lumefantrine recommended in national essential drug list as well as in health policy in the healthcare facilities in Kenya was reported for several weeks [6]. Similar availability problems have been experienced in sub-Saharan Africa [7, 8]. Prescribing inappropriate alternatives, due to shortage of recommended anti-malarial drugs, was seen as a common practice in the healthcare facilities in Uganda [9]. Delayed procurement process was held responsible for the shortage of anti-malarial drugs, and the need of addressing the current shortcomings facing antimalarial drug supply to the public sector by the national ministries of health and the international community was emphasized in Kenya [6]. 

Malaria continues to be a major public health problem in Pakistan. The total number of confirmed cases of malaria reported in 2011, in Pakistan (public sector), from all the districts was 319,592, out of which 205,879 (67%) cases were due to *P. vivax* infection, while 113,713 (33%) were due to *P. falciparum* infection. The actual malaria burden could be considered four to five times higher as nearly 70–80% of the population goes to private sector for treatment; and therefore, those malaria cases are not reported [10]. National treatment guidelines for malaria were designed and published in 2005 through collaborative efforts of directorate of malaria control, WHO, technical core group, and professionals from teaching institutions in Pakistan [11]. The guidelines have been formulated through an extensive deliberation and local research carried out by renowned professionals, malariologists, and clinicians. The policy of the National Malaria Control Program of Pakistan clearly indicates examining patients with fever microscopically or RDT kits especially children and patients with parasitemia should be treated. But due to lack of resources, technical experts, and surveillance system, microscopic diagnosis of parasitemia is usually not viable in the country. In this situation, utilization of a more specific clinical algorithm helps to diagnose accurately which assumes that when 90% of the treated patients do not have the disease and are better served by greater attention to alternative diagnosis and the prevention of overtreatment [10]. However, the positive predictive value of the algorithm remained quite low at 10% for an individual patient. Thus, even with an improved algorithm, healthcare workers should think about an alternative diagnosis, and policy makers should consider increasing the capacity for microscopic diagnosis [10].

The article "Why Hospital Pharmacists Have Failed to Manage Antimalarial Drugs Stock-Outs in Pakistan? A Qualitative Insight" was published in 2013. Journal: Malar Res Treat.

Chloroquine is the first choice of drugs for empirical therapy in all cases of malaria when type is not confirmed through laboratory test. The treatment for malaria caused by *Plasmodium vivax* includes chloroquine plus primaquine, while artesunate plus sulphadoxine/pyrimethamine is recommended for the treatment of malaria caused by *Plasmodium falciparum* [12]. However, ACT (artemether + lumefantrine) should only be administered in confirmed cases of *P. falciparum*. Malaria Control Program is functional in the country but is confined to limited districts due to financial constraints and more focused at primary healthcare facilities. Diagnostic kits and medicines, for example, chloroquine-fansidar and artemisinin combination therapy ACT, are provided free of cost in the selected healthcare facilities in targeted districts. The national standard treatment guidelines are present but are rarely followed at healthcare facilities in Pakistan which reflects weak policy implementation by the Malaria Control Program. Malaria Control Program has planned proper coordination between the public and private sector in the next five years to improve coverage for better diagnosis and treatment practices for malaria at tertiary and secondary healthcare facilities in Pakistan [13].

Effective medicine can be practiced only where there is efficient drug management. The role of pharmacists in the procurement team is vital. They are qualified professionals who follow the principles of quality assurance [14]. They realize the particulars of the distribution chain and principles of efficient stock keeping and stock turnovers. They are familiar with the pricing configuration and technical information related to drug products available within the markets [15]. They act as an interface with clinical staff to ensure that all the medicines are available to the patients through the use of appropriate stock management systems and dispensing software [16, 17]. On the other hand, hospital pharmacists have concerns about their present professional roles and face considerable barriers with regard to the provision of quality clinically focused pharmacy services in Pakistan [18]. They are more confined to traditional duties rather than patient-orientated pharmaceutical care. Their current role is more focused on pharmacy recordkeeping and is rarely involved in patient education pertaining to drugs. Although the pharmacist is part of the Drug and Therapeutic Committee, but is seldom involved in updating hospital's drug formulary [19]. Limited budget is allocated to healthcare especially for drug procurement in Pakistan like many other developing countries. Therefore, it is imperative to optimize expenditures for drug purchases through appropriate selection and procurement techniques ensuring the availability of key drugs from essential drug list for promoting the rational use of drugs. The responsibility of regulating drug prices lies with the Federal Ministry of Health. Open tender is placed through the Ministry of Health for procurement in the public sector while drugs are directly purchased from the vendors in the private sector. It is the responsibility of the Drug and Therapeutic Committee to ensure the availability of drugs in the healthcare facility in accordance with the standard treatment guidelines, but generally this is not taken into account. Therefore, the main objective of the present study was to investigate hospital pharmacists' perceptions towards factors underlying irrational treatment practices, ineffective drug management, and stock-outs of anti-malarial drugs in the two cities of Pakistan: Islamabad (national capital) and Rawalpindi (twin city).

The article "Why Hospital Pharmacists Have Failed to Manage Antimalarial Drugs Stock-Outs in Pakistan? A Qualitative Insight" was published in 2013. Journal: Malar Res Treat.

## 2. Methods

### 2.1. Study Design

A qualitative study was designed to explore the perceptions of hospital pharmacists regarding current treatment practices for malaria and responsible factors, role of healthcare system and Malaria Control Program, role of hospital pharmacist in effective drug management and influencing factors, current scenario and responsible factors of anti-malarial drugs stock-outs, and strategies to improve current practices and anti-malarial drugs stock-outs. The study protocol was approved by Malaria Control Program, Ministry of Health, Government of Pakistan. Semistructured interviews were conducted using in-depth interview guides to collect the data.

### 2.2. Participants

The study participants were hospital pharmacists working in all the tertiary healthcare facilities. The sampling frame was comprised of professionally qualified pharmacists working in both public and private tertiary healthcare facilities in two cities of Pakistan: Islamabad (national capital) and Rawalpindi (twin city).

#### 2.2.1. Sample Size and Sampling Technique

Sixteen pharmacists took part in the study. Nonprobability sampling technique, that is, snowball sampling, was adopted. Snowball sampling is the best way to identify respondents with certain attributes or characteristics and is influential in population which is difficult to contact [20, 21]. The researcher identifies the first respondent in snowball sampling, and then the respondent is asked to suggest more research participants.

### 2.3. Study Tool

A semistructured interview guide was developed after extensive literature review and used as the study tool. A number of aspects to be addressed were already identified from the literature which ensured the inclusion of key issues regarding effective drug management and stock-outs in treatment of malaria. While designing the questions, the focus was to keep them as open as possible to interviewees for maximum opportunity to express their views. The first draft of the interview guide was discussed among the authors and was modified after few rounds of discussion. The pretesting of the interview guide was carried out with eight hospital pharmacists to check whether particular questions were useful in the retrieval of information. Specific probes were identified during the pilot interviews, and the interview guide was subsequently modified. Semistructured one-to-one interviews were conducted since it is the most practical and convenient way for busy professionals, and thematic saturation was considered to be a cut-off point to stop the sampling of subjects [22].

### 2.4. Procedure and Interview Process

All the interviews were conducted from June to July 2011, at the offices of the respondents. Sixteen respondents via snowball sampling technique were recruited from tertiary healthcare facilities in Islamabad and Rawalpindi, Pakistan. Data collection was stopped at a point when no new themes emerged [22]. The identified participants were contacted in person or on phone to fix interview appointments. Written consent was obtained from each of the participants prior to the conduction of interview. Probing questions were used where necessary, and participants were given freedom to express their views at the end of the interview session. Each interview lasted approximately twenty to thirty minutes. All the interviews were conducted in the local language and at time convenient for the respondents. Permission for recording was obtained and all the interviews were recorded. Each interview was transcribed verbatim. Transcribed interviews were subjected to thematic content analysis, and the transcripts were analyzed for relevant content to identify the emerging categories [22].

The article "Why Hospital Pharmacists Have Failed to Manage Antimalarial Drugs Stock-Outs in Pakistan? A Qualitative Insight" was published in 2013. Journal: Malar Res Treat.

## 3. Results

Most of the respondents were males and had B.Pharmacy qualification. Half of the respondents were working in public tertiary healthcare facilities while the other half were employed in private tertiary healthcare facilities as hospital pharmacists.  Table 1 shows detail demographics of the respondents.

*Themes*

*Theme 1: Prevalence of Malaria in Pakistan.* Malaria was identified as a seasonal disease most frequently reported in the rainy season. *Plasmodium vivax* and *Plasmodium falciparum* were the common types of malaria observed in Pakistan stated by all the pharmacists.

*Exact statistics of malaria cases are not available in the country but it is reported more frequently in rainy season. P. falciparum and P. vivax are common types of malaria in the region. (Pharm.06)*

*Malarial cases are reported seasonally but they are also seen on and off, over the year. Falciparum and vivax are common types of malaria in Pakistan. (Pharm.01)*

*Theme 2: Current Scenario of Treatment Practices for Malaria. *All the respondents agreed that due to inappropriate diagnosis and undue recommendation of medicines on the basis of empirical therapy malaria is treated irrationally in both public and private healthcare facilities in Pakistan.

*Basically malaria diagnosis is confused with typhoid which leads to irrational treatment practices by the prescribers. (Pharm.13)*

*I feel that the treatment offered for malaria is irrational which is mostly due to inappropriate diagnosis and undue recommendation of medicines on the basis of empirical therapy. (Pharm.10)*

*Theme 3: Major Contributing Factors towards Irrational Treatment Practices for Malaria.* In view of most of the pharmacist's inappropriate diagnosis, irrational prescribing practices, unavailability of drugs, and lack of awareness of prescribers regarding standard treatment guidelines and self-medication are the major factors promoting irrational treatment of malaria in Pakistan.

*Empirical therapy is a common trend in malaria, a cocktail of anti-malarial, antibiotics and anti pyretic is presented to patient without confirmation through laboratory investigations that whether the patient is suffering from malaria or not. Besides this self medication is another major issue promoting irrational practices. (Pharm.09)*

*I think influence of pharmaceutical industry on prescribers, inadequate knowledge of prescribers and major stock-outs of anti-malarial drugs are the major factors promoting irrational treatment practices. (Pharm.04)*

*I think peer influence and unfortunately lack of training of prescribers are the major contributing factors towards irrational practices. (Pharm.11)*

*Theme 4: Role of Healthcare System in Effective Drug Management and Treatment Practices for Malaria.* Almost all the respondents were of the view that the healthcare system has failed to play a positive role in promoting rational treatment of malaria in Pakistan, but still public sector is comparatively more rational in their practices as compared to the private sector.

The article "Why Hospital Pharmacists Have Failed to Manage Antimalarial Drugs Stock-Outs in Pakistan? A Qualitative Insight" was published in 2013. Journal: Malar Res Treat.

*Public sector is more rational in their practice due to limitations in their drug lists. Private sector is more market driven and people believe that costly medicines are the only effective treatment due to which practices in the private sector is more irrational, uncontrolled, less hindered and more frequent. However, perception is different as patient is more satisfied with the private sector due to better interaction and more frequent counseling. I think the public sector is over utilized and average interaction of the physician in the public sector is less than 90 seconds. Due to less space and heavy load of patient, physicians have little time for interaction and rationality is at times compromised. (Pharm.01)*

*I think both sectors are equally involved in irrational practices but public sector is comparatively better, as prescribers and administration is not biased in the public sector due to limitations in prescribing with only available drugs in the hospital. (Pharm.09)*

*Theme 5: Role of Hospital Pharmacist in Drug Management in Pakistan.* Although the pharmacist is part of Drug and Therapeutic Committee in both public and private healthcare facilities in Pakistan, he/she has no significant role in drug selection, and procurement was stated by all the pharmacists working in public and private sector.

*Physicians can prescribe the medicine, but its selection, quality and appropriate storage needs to be channeled through the pharmacist. But due to financial constraints there are few posts of pharmacists in public sector hospitals and unfortunately the role of the pharmacist is being played by the physicians. (Pharm.01)*

*Pharmacist has a key role in drug management in the hospital but I don't see any pharmacist been involved in drug selection and procurement in public or private healthcare facilities in Pakistan. Although he/she is part of Drug & Therapeutic Committee. (Pharm.07)*

*Theme 6: Factors Underlying Inadequate Role of Hospital Pharmacist in Effective Drug Management.* All the respondents agreed that role of hospital pharmacists has not been accepted yet in Pakistan. Reluctance from physicians, unawareness of public regarding role of pharmacist, political reasons, and lower incentives were the factors responsible for inadequate role of pharmacist in effective drug management.  Table 2 shows factors underlying inadequate role of hospital pharmacist in effective drug management.

The article "Why Hospital Pharmacists Have Failed to Manage Antimalarial Drugs Stock-Outs in Pakistan? A Qualitative Insight" was published in 2013. Journal: Malar Res Treat.

*I don't think pharmacist is playing his/her clinical role effectively. The major reasons are reluctance from physicians, unawareness of public regarding role of pharmacist and lower incentives for hospital pharmacists. (Pharm.12)*

*Pharmacist has a key role in drug management in the hospital but I don't see any clinical role performed by him/her. This is mostly due to political reasons faced by the pharmacists and reluctance of physicians to involve them in drug selection. (Pharm.05)*

*Theme 7: Collaborative Working of Physicians and Pharmacists in Pakistan.* Nearly all of the respondents were of the view that there is no collaborative working of physicians and pharmacists in Pakistan, but it can promote rational treatment of malaria.

*I don't see any collaborative working of physicians and pharmacist up till now, but if it happens, it will definitely help physicians in prescribing and pharmacists in purchasing and ultimately services to the patient will improve. (Pharm.03)*

*I don't see any collaboration of physicians and pharmacists. This might be due the fact that physicians feel reluctant to accept the role of pharmacists and feel professional threat from them. (Pharm.08)*

*I think collaborative working is not there but it must be promoted and role of pharmacist must be accepted. (Pharm.05)*

*Theme 8: Role of Malaria Control Program (MCP).* All the pharmacists agreed that Malaria Control Program has failed to play its role effectively in promoting rational treatment practices and control of malaria in Pakistan.

*I think if MCP has played any role then malaria would not been the worst problem of the country. (Pharm.15)*

*No, the Malaria control program is not playing any effective role at all. I see the program as a failure. (Pharm.16)*

*MCP has a very influential role in control and promotion of rational practices for the treatment of malaria but I haven't seen their role has been justified. (Pharm.09)*

*Theme 9: Drug Management of Antimalarial Drugs in the Healthcare Facilities.* Drugs are selected on the basis of hospital formulary and quantified on the basis of consumption data in both sectors. Drugs are procured annually through open tender system and distributed on the basis of First Expired, First Out (FEFO) in the hospitals and inventory, and expiry of drugs is managed manually. On the other hand, drugs are procured quarterly through direct negotiation with the vendors and distributed on the basis of First Expired, First Out (FEFO) in the hospitals. Expiry of drugs and inventory control is done through computerized system. Same drug management procedures were performed for anti-malarial drugs in both sectors.

*(a) Role of Essential Drug List (EDL) in Drugs Selection*

*I think Essential Drug List (EDL) should be followed for drug selection but I see major issues in its up gradation and legal implementation in both sectors. (Pharm.05)*

*Due to financial constraints formulary is followed instead of Essential Drug List (EDL) for drug selection in both sectors. (Pharm.09)*

*(b) Procurement and Distribution*

*In the public sector, drugs are procured annually on the basis of consumption data and list is sent to the physicians for their feedback. They have full freedom of addition or deletion, the list is then reviewed and finalized. Open tender is placed through the Ministry of Health for procurement. Drugs are distributed on the basis of First Expired First Out (FEFO). (Pharm.01)*

*Well, we usually procure drugs quarterly on the basis of consumption data and mostly referred by the physicians in the private hospitals. Drugs are directly purchased from the vendors and distributed on the basis of First Expired First Out (FEFO) in the hospital. (Pharm.04)*

*(c) Inventory Control*

*Ledgers and books are maintained for inventory control. Triple audit and internal audit systems support our inventory management. And you will be happily surprised that not a single query has been raised against data entry and inventory management. We are absolutely clear that digitalization is the way through which we can improve the tracking of medicines easily from store to the patient, as it is very difficult to trace manually. But financial constraints are the major hurdles in doing so in the public sector. But we are looking forward for public private collaboration to achieve this. (Pharm.15)*

*Inventory list is properly updated and reviewed through the computerized system to ensure the availability of drugs in the private sector. (Pharm.14)*

*(d) Drugs Expiry Management*

*Drugs expiry is usually managed through computerized system in the private sector. The system intimate before six month to expiry as alarms are set, so usually drugs are not expired. But if in case, if due to some technical faults in the computerized system, drug expiry has been neglected, then expired drugs are discarded in front of manufacturer and drug inspectors. (Pharm.06)*

*Hospital team regularly checks the expiry of drug manually in the public sector and expiry is intimated before six month so drug expiry rarely happens. In case if drug expire then the hospital team discard the drugs in front of the drug inspector and manufacturer. (Pharm.08)*

*(e) Dispensing and Patient Counseling*

*Medication dispensing is mostly done by dispensers and counseling is not performed due to inadequate number of hospital pharmacists in the public healthcare facilities. (Pharm.10)*

*Although medicines are dispensed by the pharmacists in the private hospitals but patient counseling is limited. (Pharm.02)*

*(f) Adverse Drug Reporting System*

*No, adverse drug reporting system is present in Pakistan as physicians do not allow doing so as this is a check on them. (Pharm.09)*

*There is no adverse drug reporting system in Pakistan and I see reluctance of prescribers in its implementation. (Pharm.10)*

*Theme 10: Current Scenario of Antimalarial Drugs Stock Outs in Healthcare Facilities.* Most of the respondents were of the view that the problem of drug stock-outs is more frequent in the public sector than in the private healthcare facilities. Drug stock-outs of chloroquine and sulfadoxine/pyrimethamine (fansidar) were more prevalent in both sectors. Financial constraints, inappropriate drug management, and inadequate funding were the reasons responsible for drug stock-outs by the respondents.  Table 3 shows reasons for antimalarial drug stockouts.

The article "Why Hospital Pharmacists Have Failed to Manage Antimalarial Drugs Stock-Outs in Pakistan? A Qualitative Insight" was published in 2013. Journal: Malar Res Treat.

*Shortage of Chloroquine and fansidar in the market are the most common examples in case of malaria, as artemether/lumefentrine is being promoted due to strong influence of pharmaceutical industry. Drug stock-outs are more prevalent in the public hospitals due to inadequate resources. (Pharm.01)*

*Unethical promotion of artemether/lumefentrine by the pharmaceutical industry is responsible for the shortage of Chloroquine and fansidar in the market. This is not only increasing cost of treatment but we are also losing an effective drug due to its over prescribing. The availability of drugs due to adequate funding is better in private sector. (Pharm.06)*

*(a) Reasons for Anti-Malarial Drugs Stock-outs*

*Lack of implementation of Essential drug List, unethical promotion of drugs by Pharmaceutical Industry and prescribing are the chief factors contributing towards anti-malarial drugs stock outs. (Pharm.11)*

*Financial constraints and inappropriate calculation of lead time are the major factors which promote anti-malarial drugs stock outs. (Pharm.14)*

*(b) Role of Generic Prescribing in Preventing Stock-outs and Promoting Rational Practices*

*If drug management is based on generics we can reduce the issue of drug stock outs. I strongly recommend that it must be implemented to abolish the monopoly of physicians and pharmaceutical industry in Pakistan. (Pharm.07)*

*I think non-proprietary name prescribing can improve the availability of drugs and current practices. But it is difficult to implement this in Pakistan, as Pharmaceutical Industry is strongly influential. (Pharm.05)*

*Theme 11: Strategies to Improve Current Malaria Practices and Antimalarial Drugs Stock-Outs.* In view of most of the respondents improved diagnostic and treatment facilities, prescribing by nonproprietary name names, training of health professionals, accepted role of hospital pharmacist in drug management, implementation of essential drug list, and standard treatment guidelines for malaria in the healthcare system are the most effective strategies to promote rational drug use and control of malaria in Pakistan.  Table 4 shows strategies to improve current malaria practices and antimalarial drug stock-outs.

*I think lab investigations must be improved to ensure appropriate diagnosis of malaria. Training of prescribers regarding proper doses of anti-malarial drugs must be conducted. Patient counseling must be ensured to limit self medication in treatment of malaria. Essential drug list and Standard Treatment Guidelines for malaria must be implemented in the country. (Pharm.04)*

*Implementation of Essential drug list and generic prescribing can improve availability of anti-malarial drugs. Training of health professionals regarding Standard Treatment Guidelines and efficient drug management can improve the current treatment practices for malaria. Clinical role of hospital pharmacist must be accepted as a healthcare team member. (Pharm.11)*

## 4. Discussion

The healthcare system has failed to play a positive role in promoting rational treatment for malaria in Pakistan. The respondents agreed that inappropriate diagnosis and undue recommendation of medicines on the basis of empirical therapy are common trends in both public and private healthcare facilities, but still the public sector is comparatively more rational in their practices as compared to the private sector. The results of the present study are in line with the study conducted in Nigeria where the use of presumptive malaria diagnosis without laboratory support was a common diagnostic procedure for malaria and inclined to poor quality of malaria diagnosis and treatment [23]. In view of most of the pharmacists' inappropriate diagnoses, irrational prescribing practices, unavailability of drugs, and lack of awareness of prescribers regarding standard treatment guidelines and self-medication are the major factors promoting irrational treatment for malaria in Pakistan. Similar patterns of irrational drug use in other countries have been reported [24, 25].

The article "Why Hospital Pharmacists Have Failed to Manage Antimalarial Drugs Stock-Outs in Pakistan? A Qualitative Insight" was published in 2013. Journal: Malar Res Treat.

All the respondents agreed that Malaria Control Program has not played its role effectively in promoting rational drug use and control of malaria in Pakistan. This might be due to the fact that Malaria Control Program has targeted mainly 19 districts in different provinces due to shortage of funds and has not been able to target tertiary and secondary healthcare facilities. However, the national malaria control programs were successful in reducing the number of malaria cases in Iran and Uganda [26].

The concept of essential drugs has been introduced in Pakistan to concentrate resources on the most cost-effective and affordable drugs to treat prevailing health problems. National Essential Drugs List of Pakistan was first prepared in 1994. The list was previously reviewed in 1995 and 2000 and has not been updated since 2007. The list contains 452 drugs of different pharmacological classes. Drug and Therapeutic Committee for procurement of drugs was placed in all the healthcare facilities. All the pharmacists working in public and private sector agreed that although the pharmacist is part of Drug and Therapeutic Committee in both public and private healthcare facilities in Pakistan, he/she has no significant role in drug selection and procurement. The clinical role of hospital pharmacists has not been accepted yet in Pakistan. Reluctance from physicians, unawareness of public regarding role of pharmacist, political reasons, and lower incentives were the factors responsible for inadequate role of pharmacist in effective drug management. This situation is quite similar in other developing countries [27]. Nearly all of the respondents were of the view that there is no collaborative working of physicians and pharmacists in Pakistan, but it can promote rational treatment of malaria. The results of the present study are in line with findings of another study which reported that interaction between the pharmacists and physicians is low in Pakistan and emphasized the need of collaboration of pharmacists with other healthcare professionals for achieving the goals of pharmaceutical care [19].

Drugs are selected on the basis of hospital formulary instead of Essential drug list and quantified on the basis of consumption data in both sectors. Drugs are procured annually through open tender system and distributed on the basis of First Expired, First Out (FEFO) in the hospitals and inventory and expiry of drugs are managed manually in the public healthcare facilities. On the other hand, drugs are procured quarterly through direct negotiation with the vendors and distributed on the basis of first expired first out (FEFO) in the hospitals. Expiry of drugs and inventory control is done through computerized system. The results of the present study are in line with another study which showed similar drug management system in different healthcare facilities in Nigeria [28].

The article "Why Hospital Pharmacists Have Failed to Manage Antimalarial Drugs Stock-Outs in Pakistan? A Qualitative Insight" was published in 2013. Journal: Malar Res Treat.

Most of the respondents were of view that the problem of drug stock-outs is more frequent in the public sector than in the private healthcare facilities. Similar results of unavailability of key antimalarial drugs in healthcare facilities were reported by several studies. Drug stock-outs of chloroquine and sulphadoxine/pyrimethamine (fansidar) were more prevalent in both sectors in Pakistan. This might be due to unethical promotion of artemether/lumefantrine by the pharmaceutical industry. Financial constraints, inappropriate drug management, and inadequate funding were the reasons responsible for drug stock-outs by the respondents. Similar factors were responsible for the unavailability of key antimalarial drugs in healthcare facilities in Kenya [6].

Improved diagnostic and treatment facilities, prescribing by nonproprietary names, training of health professionals, accepted role of hospital pharmacist in drug management, and implementation of essential drug list and standard treatment guidelines for malaria in the healthcare system were stated as the most effective strategies by the respondents to promote rational drug use and control of malaria in Pakistan. Various intervention studies have reported significant impact on diagnostic and treatment practices [29, 30].

*Limitation of the Study.* The study was conducted in the two cities of Pakistan. It is most likely that the health practitioners in other parts of the country would have similar perceptions regarding treatment practices carried for malaria, but the findings may not be generalizable to the other cities of the country. 

## 5. Conclusion

Based on the results of this qualitative study, all the pharmacists agreed that irrational prescribing practices, ineffective drug management, lack of implementation of essential drug list, and problem of anti-malarial drugs stock-outs are the major factors contributing towards irrational treatment practices for malaria in both public and private sectors in Pakistan. Hospital pharmacists have failed to play an effective role in the efficient management of anti-malarial drugs stock-outs. Reluctance from physicians, unawareness of public regarding role of pharmacist, political reasons, strong influence of pharmaceutical industry, and lower incentives are the factors responsible for this inadequate role of pharmacist. Innovative approaches are needed to allocate funds for the public sector through collaborative working with the private sector, implementation of national essential medicine list in all the healthcare facilities, and promotion of nonproprietary name prescribing to ensure the availability of drugs. For effective drug management and improved pharmaceutical care services, the role of the pharmacist as an integral member of healthcare team has to be accepted by the stakeholders, health professionals, and community in Pakistan.

The article "Why Hospital Pharmacists Have Failed to Manage Antimalarial Drugs Stock-Outs in Pakistan? A Qualitative Insight" was published in 2013. Journal: Malar Res Treat.

## Figures and Tables

**Table 1:** Demographic characteristics of pharmacists.

Code	Gender	Qualification	Experience	Sector	Current designation
Pharm. 1	Male	B.Pharmacy	10 years	Public	Hospital pharmacist
Pharm. 2	Male	Pharm.D	3 years	Private	Hospital pharmacist
Pharm. 3	Female	B.Pharmacy, MBA	2 years	Public	Hospital pharmacist
Pharm. 4	Male	MPhil.Pharmacy	14 years	Private	Hospital pharmacist
Pharm. 5	Female	B.Pharmacy	9 years	Public	Hospital pharmacist
Pharm. 6	Male	Pharm.D	2 years	Private	Hospital pharmacist
Pharm. 7	Female	B.Pharmacy	4 years	Public	Hospital pharmacist
Pharm. 8	Male	MPhil.Pharmacy	9 years	Public	Hospital pharmacist
Pharm. 9	Male	B.Pharmacy	1 years	Private	Hospital pharmacist
Pharm. 10	Male	Pharm.D	10 years	Public	Hospital pharmacist
Pharm. 11	Female	B.Pharmacy	17 years	Private	Hospital pharmacist
Pharm. 12	Male	B.Pharmacy	14 years	Private	Hospital pharmacist
Pharm. 13	Male	B.Pharmacy	6 years	Private	Hospital pharmacist
Pharm. 14	Male	Pharm.D	2 years	Private	Hospital pharmacist
Pharm. 15	Male	B.Pharmacy	17 years	Public	Hospital pharmacist
Pharm. 16	Female	Pharm.D	7 years	Public	Hospital pharmacist

Pharm.: Pharmacist, B.Pharmacy: Bachelors in pharmacy, Pharm.D: Doctor of pharmacy, Mphil: Master of Philosophy, and MBA: Masters of Business Administration.

**Table 2:** Factors underlying inadequate role of hospital pharmacists in effective drug management.

Variable	*n* (%)
Reluctance from physicians	14 (87.5)
Unawareness of public regarding the role of the pharmacist	9 (56.2)
Lower incentives	15 (93.7)
Political reasons	8 (50)

**Table 3:** Reasons for anti-malarial drugs stock-outs.

Variable	*n* (%)
Lack of implementation of essential drug list	15 (93.7)
Unethical promotion of drugs by pharmaceutical industry	10 (62.5)
Financial constraints	15 (93.7)
Prescribing practices	14 (87.5)
Inappropriate calculation of lead time	12 (75)
Lack of generic prescribing	9 (56.2)

The article "Why Hospital Pharmacists Have Failed to Manage Antimalarial Drugs Stock-Outs in Pakistan? A Qualitative Insight" was published in 2013. Journal: Malar Res Treat.

**Table 4:** Strategies to improve anti-malarial drugs stock-outs.

Variable	*n* (%)
Implementation of essential drug list and standard treatment guidelines	14 (87.5)
Acceptance of role of hospital pharmacist	15 (93.7)
Improved availability of anti-malarial drugs	11 (68.7)
Efficient drug management	14 (87.5)
